The article "Risk Management of Sports Venues and Olympic Sports Cooperation Spirit under Complex Environment" was retracted in 2023. Reasons: signs of a paper mill; suspected computer-generated content; unreliable results or conclusions; lack of ethics approval or compliance.

# Risk Management of Sports Venues and Olympic Sports Cooperation Spirit under Complex Environment

**DOI:** 10.1155/2022/9127539

**Published:** 2022-08-31

**Authors:** Dianzai Jiang

**Affiliations:** Fujian Business University, FuZhou 350000, China

## Abstract

The understanding of sports event risk and Olympic sports cooperation spirit, as well as the systematic analysis and research of sports event risk management, are still in their early stages in China's sports theory circle. Institutions for developing sports talent also disregard programmes designed to increase the risk awareness and Olympic spirit of sports workers. This essay provides an overview of the concepts of sports event risk and Olympic sports cooperation spirit based on reality. This paper examines the interaction of risk management of large-scale sporting events and Olympic sports cooperation spirit from the perspective of event organization managers, using the pertinent theory of risk management and the random forest algorithm in machine learning. The experimental results show that, according to the analysis of injury occurrence according to different positions, it is discovered that forward athletes suffer the most injuries, with an average of 54 forwards in injury situations, followed by guards with an average of 43 guards in injury situations, and finally centres with an average of 38 guards in injury situations. Combining risk management for major sporting events with the cooperative Olympic sports spirit has significant practical implications.

## 1. Introduction

With the development of sports in China, sports exchanges between China and other countries are increasing, and many cities in China are undertaking large-scale sports events at home and abroad. With the continuous expansion of the scale of sports events, all kinds of uncertain factors in sports events increase the risk of sports events. However, in China's sports theory circle, the understanding of sports event risk and Olympic sports cooperation spirit and the systematic analysis and research of sports event risk management are still in the primary stage, and the sports talent training institutions also neglect the training of sports workers' risk awareness and Olympic sports cooperation spirit [1]. The risk management of the competition refers to the possible interruption, delay, and cancellation of the competition due to the low level of planning and maintenance or negligence during the operation of the competition. During a series of operations before, during, and after a large-scale sports event, the objectivity and uncertainty of its risks are inherent in the event itself. At the same time, the continuous commercialization of the operation mode of the competition and the continuous clarification of the property rights related to the competition make the competition-related subjects have to be responsible for their own profits and losses, and become the risk-taking subjects, thus making the competition risk management and the Olympic sports cooperation spirit necessary [2, 3]. The introduction of risk management is not to increase the operation cost of sports events, but to reduce all kinds of uncertain damaging factors in the process of holding sports events, so as to increase the reliability and stability of the benefits of holding sports events. However, in the operation of sports events, risk management and Olympic sports cooperation spirit are still in a spontaneous, perceptual and empirical stage, which is extremely out of proportion with the progress of society and the development of sports events themselves. Therefore, it is necessary to strengthen the research on risk management of sports events and Olympic sports cooperation spirit, strengthen the ability of risk management of sports events and Olympic sports cooperation spirit and provide guarantee for the successful operation of sports events [4].

The article "Risk Management of Sports Venues and Olympic Sports Cooperation Spirit under Complex Environment" was retracted in 2023. Reasons: signs of a paper mill; suspected computer-generated content; unreliable results or conclusions; lack of ethics approval or compliance.

This paper provides a summary of the concepts of sports event risk and Olympic sports cooperation spirit starting from the reality. It investigates the interaction of risk management of large-scale sporting events and Olympic sports cooperation spirit by utilizing related theories of risk management and the random forest algorithm in machine learning. The term “random decision trees” also refers to the many decision trees that make up the random forest [5, 6]. The trees in the random forest have no relationship to one another. The decision tree used to classify the test data when it enters the random forest is actually used as the final result; it is the one with the greatest number of classification successes across all decision trees. The random forest algorithm not only achieves high recognition accuracy but also time effectiveness, making it more suitable for practical production and application. It even has good image extraction capabilities for radar and other types of images. Because it is more effective than other machine learning techniques as well as conventional statistical methods, the random forest classification method is appropriate for the classification of images using a variety of data types and classification systems. The random forest algorithm's general procedure is to identify the tree with the highest information benefit in attribute set A, choose it as the root node, divide the sample set into all subsets based on the value of the root node's attribute, remove this attribute from the attribute set, and then choose the attribute with the highest information gain value in each subset as the current subset's root node and the child node of the upper set's root node, if each of the sample attributes in the subset that was obtained falls into a single category [7, 8]. The classification process's deviation is dependent on how well each tree performs and how similar the trees are to one another in the random forest algorithm, which uses trees with identical distribution structures. Each node in the feature selection process is divided randomly, and the errors in various scenarios are then compared.

The article "Risk Management of Sports Venues and Olympic Sports Cooperation Spirit under Complex Environment" was retracted in 2023. Reasons: signs of a paper mill; suspected computer-generated content; unreliable results or conclusions; lack of ethics approval or compliance.

By analyzing and exploring the definition, characteristics and operation methods of sports event risk management and Olympic sports cooperation spirit, and summarizing the successful and unsuccessful experiences of competition risk management at home and abroad, this paper puts forward a set of operation modes suitable for China's sports event risk management, improves the risk management awareness of the event organizers, serves all kinds of sports events in China and lays a theoretical foundation for the theoretical research of Olympic sports cooperation spirit [9]. On the basis of transforming athletes' three-dimensional acceleration data into discrete binary data, the forest algorithm needs to automatically classify athletes' activities by using the classifier in machine learning. Finding a more accurate and efficient classifier can enhance the success rate of the injury possibility monitoring system. It can be said that the reputation of the Olympic Movement is inseparable from modern media. The spread of the Olympic Movement and modern media technology interact, promote and rely on each other. In the process of spreading, the Olympic spirit and culture are also spread accordingly [10, 11]. Therefore, it is essential to implement a variety of efficient risk management strategies using the random forest algorithm to lower the likelihood of risk accidents and the harm they cause, in order to foster the spirit of cooperation between the Olympic sports and the games and further the industrialization and marketization of sports. Combining risk management for major sporting events with the cooperative Olympic sports spirit has significant practical implications.

I put forward the following innovations in this paper: (1) The decision tree of the proposed random forest algorithm is discussed, as well as the algorithm itself. Selecting the attribute splitting on the tree's nodes in order to choose the best attribute selection is the main challenge of the decision tree algorithm. Results for classification can vary depending on the attribute selection rules used. The number of information bribes is used to determine the various nodes at each level of the decision tree, that is, the crucial characteristics for classification, in order to solve this problem. The growth process of a decision tree is the procedure used to create a decision tree using continuous layering from the training sample set. Many different branches are also created during this process. (2) There has been investigation, design and implementation of the research on the construction of the discourse power of Marxist ideology. The conflicts and contradictions between various ideologies are escalating as a result of the big data revolution's quick spread and integration as well as its influence on public discourse. We must actively use new media to interpret and quickly disseminate the most recent theoretical developments of Marxism in China in order to achieve short-term, all-around success. We must also be vigilant against the ideological infiltration of capitalist countries for the purposes of “Westernization” and “differentiation.” By spreading Marxist ideology in three dimensions, the general populace will be better equipped to fend off diverse ideologies and defend the fundamentals of Marxism.

The article "Risk Management of Sports Venues and Olympic Sports Cooperation Spirit under Complex Environment" was retracted in 2023. Reasons: signs of a paper mill; suspected computer-generated content; unreliable results or conclusions; lack of ethics approval or compliance.

## 2. Related Work

The risks faced by large-scale sports events in the course of operation are more complicated, and various uncertain factors in the events increase in line with the increase in the number of large-scale sports events in China, the expanding scale and influence and the changing environment of the events. It is necessary to carry out risk management of sporting events, which should be put on the agenda. With the commercialization of the operation mode of contemporary sporting events and the clarification of the property rights associated with the events, the main body of event management must be accountable for its own profits and losses and become the main body of risk. The implementation of risk management at sporting events is beneficial to the events' smooth progression and the realization of their advantages. As a result, this has been the subject of research by numerous academics.

Luan pointed out that the characteristics of large-scale sports events and the expansion of their scale lead to an increase in the probability of risk events. The probability of the occurrence of the risk increases, so it is very important to manage the risk of the event [12]. Ba pointed out that before a large-scale sports competition, the organizing committee of the competition must set up a risk management organization composed of experts in risk management, which is mainly responsible for all risk management matters from the preparation to the holding stage of the competition. According to the needs of the competition, several groups can be set up in the risk management institution, and the institution setting should be flat as far as possible, which can improve the work efficiency of the whole organization [13]. Shobana and Suguna show that the operation process of major sports events is complicated, involving many departments, and the risks exist in all stages and departments of the event operation, and the risks of various departments are mutually influenced and implicated, which requires all members involved in the event operation to undertake certain risk management responsibilities and cooperate with each other [14]. In order to ensure the success of sports competitions, Gao and Kowalczyk identify and evaluate various risks that may arise during the planning and holding of sporting events. Based on their findings, they then optimize and combine different risk management technologies to effectively control these risks and handle the fallout from losses brought on by these risks [15]. The argument made by Krishna et al. is that contemporary sporting events can no longer be adequately served by empirical risk management behaviour. In order to manage risk at sporting events using more sophisticated technologies and scientific methods, it is essential to implement a systematic risk management theory [16]. This will ensure the success of sporting events. Groll et al. show that the probability of risk occurrence in the process of competition organization is far greater than that of general sports activities, and the level of risk hazards is far higher than that of general sports activities. The organization and management of large-scale sports events is a very complicated and huge systematic project, which specifically involves the arrangement of competition venues, schedule, time schedule, etc., and these arrangements, together with transportation, information and communication, safety facilities, weather conditions and cultural facilities, form a complex dynamic system. Any problem in any link will seriously affect the smooth holding of sports events [17]. Zhao et al. analyze the external environment of the competition, analyze the technology, personnel, equipment and other factors involved in every link of the whole management process and operation process of the competition, and describe the risk characteristics and determine which risk events may affect the competition. Risk identification methods include work breakdown structure method, brainstorming method and interview method [18]. Xiu-Mei put forward that no special risk management organization has been set up for sports events, and there are no special risk management personnel to organize and coordinate the risks of the whole event. All departments of sports events are still “divided and guarded by troops,” and when problems arise, all departments often fail to coordinate and command in time, so that the risk events are extended to other departments, resulting in greater losses [19]. Ainsworth and Sallis pointed out that with the continuous expansion of the scale of modern sports events, various complicated and difficult-to-accurately grasped factors in the events also increased, which increased the probability of event risks to a certain extent [20]. SOA puts forward that this risk prevention behaviour in the operation of sports events in China is still in a spontaneous, perceptual and empirical stage, and has not risen to the theoretical level of risk management [21].

The article "Risk Management of Sports Venues and Olympic Sports Cooperation Spirit under Complex Environment" was retracted in 2023. Reasons: signs of a paper mill; suspected computer-generated content; unreliable results or conclusions; lack of ethics approval or compliance.

In this paper, the combination of risk management in sports venues and the spirit of Olympic sports cooperation is studied. Using the random forest algorithm in machine learning and wearable monitoring equipment, a monitoring system for athletes' injury possibility with high accuracy and low overall cost is constructed. There are many factors that affect the successful operation of the competition, such as the main factors of the competition, such as the staff, spectators, athletes and officials of various countries, the external factors such as politics, economy, culture and environment when the competition is held, the material factors such as venues and facilities, equipment and other material factors, and the humanistic factors such as the operation and management experience of the organizers of the competition, which may induce the competition risk. Through the random forest algorithm's investigation of the event managers, most people think that there are risks in the operation of sports events, and acknowledge the important role of risk management. However, some sports teams are still lucky, thinking that the probability of risk is basically zero. Athletes' physical foundation cannot better bear the required amount of exercise during competition and training, lack the means to prevent sports injuries, and treat the sports injuries in time or improperly: in the random forest algorithm, the physical resistance to collision, opponent's foul, take-off and fall, improper technical action methods and so on. Establish the concept of “service,” that is, how many risks are identified, so as to prevent the occurrence of risk events and satisfy the audience. At the same time, to improve the random forest algorithm, the concept of service should be set up within each department of sports events, and the risk management department should make a service gesture to ensure the smooth progress of each department's work and the whole event.

The article "Risk Management of Sports Venues and Olympic Sports Cooperation Spirit under Complex Environment" was retracted in 2023. Reasons: signs of a paper mill; suspected computer-generated content; unreliable results or conclusions; lack of ethics approval or compliance.

## 3. Method

### 3.1. Principles and Advantages of Random Forest Algorithm

A specific subset of statistical learning theory is represented by the random forest algorithm. The random forest forms K classification trees in accordance with the self-help sample data set to create a combination after using the bootstrap resampling method to randomly select a group of new learning samples from the initial learning sample set n. Each combination decision tree must vote on the algorithm's classification results. The algorithm's prediction result has received the most votes in this category. Its main objective is to improve the decision tree classification algorithm, which combines various decision trees. Each tree's growth is dependent on its growth from samples that were independently chosen at random [22]. Numerous fields have used random forest because of its benefits. In this chapter, decision trees' fundamentals are covered along with the random forest construction process. We can understand random forest algorithm optimization through an analysis of fundamental knowledge.

The decision trees used in the random forest algorithm are numerous. A decision tree is a type of tree structure that can have either a binary or nonbinary tree structure. The test of a feature on attributes is represented by all nonleaf nodes in the tree structure. The attribute of this feature is the output of each branch of the decision tree on a set of values, and each leaf node in the tree will store a category. Although each tree's capacity for classification may be quite small, after a large number of decision trees have been generated at random, test samples can choose the attributes for the most categories by statistically examining each tree's capacity for classification [23]. The main challenge of the decision tree algorithm is to choose the best attribute selection by choosing the best attribute splitting on the tree's nodes. Different classification outcomes can be found using various attribute selection rules. We introduce the idea of information gambling to address this issue and use the quantity of information bribes to identify the various nodes at each level of the decision tree, or the crucial characteristics for classification. The decision tree is created through continuous layering from the training sample set during the decision tree growth process. Various branches are also formed during this process. The decision tree's growth will come to an end if grouping any more groups of data makes no sense, at which point all of the branches corresponding to those groups of data will stop expanding. A complete decision tree is produced at this point. The key to decision tree growth is therefore how to establish the branching criteria. The schematic diagram of the decision tree growth process is shown in Figure 1.

The article "Risk Management of Sports Venues and Olympic Sports Cooperation Spirit under Complex Environment" was retracted in 2023. Reasons: signs of a paper mill; suspected computer-generated content; unreliable results or conclusions; lack of ethics approval or compliance.

The advantage of forest algorithm itself is mainly because it uses two random variables, one is the random extraction of features, the other is the random extraction of samples. The general principle of reaching leaf nodes is that the output variables of the samples in the nodes are of the same category or meet the standard of stopping growth specified by the user. When determining the best grouping variables, data input variables need to be grouped, and the heterogeneity of output variables can be judged by variance. Its mathematical definition is

(1) $$\begin{array}{c} R_{t}=\frac{1}{Nt-1}\sum_{i=1}^{N_{t}}, \end{array}$$

where *t* is the node and *N*_*t*_ is the sample size contained in the node *t*.

The decreasing degree of heterogeneity is measured by the decreasing amount of variance, which is mathematically defined as

(2) $$\begin{array}{c} \Delta R_{t}=R_{t}-\frac{N_{r}}{N}R_{tr}, \end{array}$$

where *R*_*t*_ and *N* represent the variance and sample size of output variables before grouping. Therefore, the observed data can be divided into two groups according to the variable and its group limit or “super class,” that is, a branch grows under the current node.

Given that {*h*_1_(*x*), *h*_2_(*x*), ...*h*_*N*_(*x*)} and *x* are input vectors and *y* is the corresponding output vector, the interval margin function of the sample point (*x*, *y*) is defined as follows:

(3) $$\begin{array}{c} mg\left(x,y\right)=avkI\left(h_{k}\left(x\right)=y\right), \end{array}$$

where *I* is the indicator function and *avk* is the average value. The interval *mg*(*x*, *y*) measures the minimum difference between the average number of votes and the classifier set classifies the *x* of a specific sample into the right category and the wrong category. The larger the interval, the better the performance of the classifier.

The generalization error of the classifier can be expressed as

(4) $$\begin{array}{c} PE=P_{X,Y}. \end{array}$$

The foot mark *X*, *Y* in the formula indicates that the probability is obtained in *X*, *Y* space.

In a random forest, *hk*(*x*)=*h*(*x*, *θ*). When the number of trees in the forest reaches a certain value, it follows the strong law of large numbers. When the number of trees increases, *PE* converges to almost everywhere for all sequences *θ*.

(5) $$\begin{array}{c} P_{X,Y}\left(P\left(h\left(x,\theta \right)\right)=y\right), \end{array}$$

where *θ* is the random vector of the single-class decision tree and *h*(*x*, *θ*) is the output of the classifier based on *x* and *θ*.

The article "Risk Management of Sports Venues and Olympic Sports Cooperation Spirit under Complex Environment" was retracted in 2023. Reasons: signs of a paper mill; suspected computer-generated content; unreliable results or conclusions; lack of ethics approval or compliance.

It shows that the generalization error of random forest always tends to the previous one with the increase of trees, and there will be no over-fitting problem.

The upper bound of random forest generalization error is

(6) $$\begin{array}{c} PE\leq \overset{-}{\rho }\left(1-s\right), \end{array}$$

where $\overset{-}{\rho }$ and *s* are the average correlation coefficient and average strength of the tree, respectively.

Random forest is an effective prediction model in machine learning algorithm [24, 25], which is an effective combination of classifier algorithm and decision tree classification algorithm. It is mainly divided into the following three advantages:

- Excellent performance of random forest classification
- The two internal random characteristics not only make the random forest have a good noise reduction effect, but also make it difficult to fall into over fitting. It has the advantage of accuracy in data set classification, and can quickly and efficiently analyse a large number of data. For example, it can process tens of thousands of unfiltered variables, and can also be used to classify uneven data sets, so as to effectively balance the error in all data.
- Random forest can provide many additional data descriptions
- It is possible to calculate the weights of each feature in the model using the random forest algorithm. By unbiasedly estimating the generalized error, a random forest model can be built to estimate the information lost in the data set. Additionally, the correlation between outlier location and cluster analysis can be estimated using the random forest model.
- Random forest has very fast computing speed
- Because all the split nodes of the tree are obtained through comparative calculation, and the operation time is positively related to the depth of each tree, the regression or classification on the tree with good performance will be fast. The operation time in the learning process of random forest algorithm is positively correlated with the number and size of trees in the model.

Random forest is based on tree classifier {*h*(*x*, *θ*_*k*_), *k*=1, ...}, in which *h*(*x*, *θ*_*k*_) is the classification regression tree that has not been pruned. *x* is an input vector, {*k*} is an independent and identically distributed random vector, and the growth process of a single tree in a random forest is determined by *k*; the final output of random forest regression is the average of the output of each single tree.

### 3.2. Construction of the Injury Possibility Monitoring System for Risk Management of Sports Venues

In recent years, large-scale sports events have become the object of competition in many countries and regions. In order to obtain the right to hold large-scale sports events, the sponsors often go all out at any cost and compete to undertake them. Therefore, sports competitions are becoming more and more frequent. The body is affected by this movement limitation and asymmetry, so that when the body performs the same movement, compensatory movements will occur in other parts of the body when the left and right sides are completed, which will reduce muscle strength, leak body energy, and increase the injury risk of athletes [26]. Sports event risk management belongs to a branch of risk management, so the mode of event risk management basically borrows from the general management mode of risk management. Experts and scholars have conducted some research on the event risk in the sports field under this framework. The development of sports must be based on certain preparatory work before it can be better carried out. It is necessary to avoid such problems as ligament injury caused by direct sports without preparatory activities. Therefore, teachers must pay attention to preparatory activities in the process of sports injury prevention. Functional movement screening can detect the movement limitation and asymmetry of the body in terms of flexibility and stability, and then improve the movement efficiency of athletes and reduce the incidence of sports injury through intervention measures. In view of this, this paper proposes a sports injury monitoring system. Sports injury monitoring is a systematic and complex process. On the basis of basically clear data processing scheme, this paper mainly investigates the possibility of sports injury in the lower leg, thigh and hip of joggers, and puts forward suggestions for the monitoring and prevention of sports injury in the knee and hip joints, so as to prove whether the random forest algorithm can be used to design athletes. The sports injury monitoring system is shown in Figure 2.

The article "Risk Management of Sports Venues and Olympic Sports Cooperation Spirit under Complex Environment" was retracted in 2023. Reasons: signs of a paper mill; suspected computer-generated content; unreliable results or conclusions; lack of ethics approval or compliance.

In the joint injury monitoring system under sports intensity training, the fuzzy theory and the grey correlation theory are combined at first. The law of joint injury under running intensity training is analyzed, the basic influencing factors of joint injury are obtained, and the expression form of the T reference sequence of fuzzy correlation analysis model of influencing factors of joint injury under intensity training is as follows:

(7) $$\begin{array}{c} Y_{t}=\left[y_{t}\left(1\right),...,y\left(k\right)\right]. \end{array}$$

In the formula, *y*_*t*_(1), ..., *y*(*k*) represents the specific description form of the *t* reference sequence in the fuzzy grey relational analysis model, which is the basic influencing factor of joint injury, and describes the periodic variation law of *y*_*t*_.

If there are *n* levels of athletes' load training intensity, the corresponding vector matrix that marks the influencing factors of joint injury under each load training intensity is as follows:

(8) $$\begin{array}{c} X_{t}=\left[x_{t}\right]=\left[x_{t}\left(1\right),...,x_{1}\left(n\right)\right], \end{array}$$

where *X*_*t*_ represents the reference sequence in the fuzzy grey correlation analysis model of influencing factors—the corresponding comparison sequence *Y*_1_.

The approximation between different joint influencing factors is judged by the cosine of the included angle of the two parameters, and the approximation matrix in the joint influencing factor analysis model is established in the following equation:

(9) $$\begin{array}{c} r_{tj}=\sum_{k=1}^{n}y_{tk}x_{jk}, \end{array}$$

where *y*_*tk*_ represents the duration of joint injury, *x*_*jk*_ represents joint activity, and *k* represents sequence points and the difference between all comparison sequences and reference sequences in the fuzzy grey correlation analysis model of joint injury influencing factors under running intensity training; then, the grey correlation model of joint injury influencing factors is

(10) $$\begin{array}{c} \xi_{tj}\left(k\right)=\left(\Delta_{\min}+\theta \Delta_{\max}\right), \end{array}$$

where *ξ*_*tj*_(*k*),  (*j*=1,2, ..., *m*) represents the correlation coefficient of different corresponding points in the reference sequence *Y*_*t*_ and the comparison sequence *X*_*t*_ in the grey correlation analysis model for the influencing factors of joint injury, and Δ_min_ represents the minimum absolute difference of all corresponding elements in *Y*_*t*_ or *X*_*t*_.

The framework of sports damage analysis consists of three core parts:

- Data processing process
- Feature extraction is carried out, and the related data is converted into binary discrete data that can be processed by computer. Then, the random forest algorithm is used as a classifier to effectively classify sports injuries, and the related data is sent to the sports injury monitoring database as the motion displacement curve that may cause sports injuries.
- Monitoring number of sports injuries
- There are injury prevention suggestions provided by sports and health experts for various possible motion displacement curves in the database. Because machine learning is a long-term process, with the continuous input of sports injury monitoring data into the database, the number of samples in the database will continue to increase, thus realizing more effective sports monitoring.
- Mechanical analysis process
- Sports injuries of athletes' lower body, knee joints and hip joints, so it is necessary to install three-axis gyroscopes in their legs, thighs and hips in wearable intelligent devices to record three-dimensional acceleration data.

The article "Risk Management of Sports Venues and Olympic Sports Cooperation Spirit under Complex Environment" was retracted in 2023. Reasons: signs of a paper mill; suspected computer-generated content; unreliable results or conclusions; lack of ethics approval or compliance.

The functional movement screening of the sports injury monitoring system can detect the limitation of the body's functional movement and the asymmetry of the body in terms of flexibility and stability. According to the test results of the sports injury monitoring system, we can formulate and design the practice means of correcting movements, so as to effectively avoid sports injuries caused by wrong movements and improve the work efficiency and rationality of sports movements. The above-mentioned research contents are applied to the empirical study of risk management of large-scale sports events, and the risk factors are analyzed. The analytic hierarchy process (AHP) is used to evaluate the risk of this event, so as to implement effective risk management for the event. In order to study the risk management of large-scale sports events qualitatively and quantitatively in the future, a beneficial exploration and attempt has been made.

## 4. Research Results and Division

### 4.1. Score Results of Motor Function Screening

According to the screening results of motor function, 63 people had a history of injury, with an average score of 15.74, a standard deviation of 2.62, a 94% confidence interval of 15.04–16.37 and a percentage of 88.55%. There were 7 persons with history of nondestructive injury, the average score was 17.12, the standard deviation was 1.25, the 94% confidence interval was 16.17–18.05 and the percentage was 11.42%, as shown in Table 1.

The experimental results showed that the sum of squares of inter-group and intra-group deviations was 13.871, 431.213, and the total sum of squares of deviations was 445.085, mean square: the mean square of inter-group was 13.871, and the mean square of intra-group was 6.342; *F* value was 2.187, significance *p* = 0.143 > 0.04. The results showed that there was no significant difference between the results of motion function screening and early injury.

According to the results of motor function screening, there were 22 subjects who showed physical asymmetry, with an average score of 17.31, a standard deviation of 1.28, a 94% confidence interval of 15.93–17.71, and a percentage of 32.85%. There were 46 people with asymmetric body, the average score was 12.95, the standard deviation was 3.42, the 95% confidence interval was 12.15–13.74 and the percentage was 67.13%, as shown in Table 2.

The article "Risk Management of Sports Venues and Olympic Sports Cooperation Spirit under Complex Environment" was retracted in 2023. Reasons: signs of a paper mill; suspected computer-generated content; unreliable results or conclusions; lack of ethics approval or compliance.

The experimental results show that the scores of symmetrical and asymmetrical subjects in the table are tested by one-way variance, and the sum of variance between groups is 27.555, the sum of variance within groups is 417.531, and the total variance is 445.085. The mean square is 27.555 between groups and 6.141 within groups. The value of *f* is 4.487, with significance *p* = 0.037 < 0.04.

In the damage analysis, the damage is divided into contact damage and noncontact damage according to different damage scenarios, and the difference between them is analyzed by paired *T* test. According to the athletes' sports grades and special positions during the competition, the injury differences of athletes among different sports grades and different special positions were compared by one-way ANOVA. In this experiment, forwards, centres and guards were used to study the injuries in different positions on the field. The experimental results are shown in Figure 3.

The experimental results show that, according to the analysis of the injury occurrence according to different positions, it is found that the injury occurrence of forward athletes is the most, the average number of forwards in the injury situation accounts for 54, followed by guards, the average number of guards in the injury situation accounts for 43, and finally the centre, the average number of guards in the injury situation accounts for 38.

In this experiment, the exposed person's times and duration of the League preparation period were studied. During the League preparation period, the training arrangement of women basketball players for one week generally includes six technical and tactical training, three physical training and one simulated competition exercise. The training participation in the preparation period is shown in Figure 4.

The experimental results show that in the 22-week follow-up record, the cumulative exposure time of athletes is 1979, and the exposure time is 5545  h hours. The average exposure was 89.95 person-times and 252.04 h hours per person, and the average exposure was 2.8 h hours per time. According to the different injury scenarios, the following table shows the athletes' injuries during the league preparation period. The team suffered an average of 3.6 injuries per week. During the whole league preparation period, injuries are mostly distributed in the first half of the league, especially from the 9th week to the 14th week. During these six weeks, the whole team suffered an average of 5.6 injuries per week. The injury can be divided into contact injury with others or objects and noncontact injury. Statistics of injury during the league preparation period are shown in Table 3.

The article "Risk Management of Sports Venues and Olympic Sports Cooperation Spirit under Complex Environment" was retracted in 2023. Reasons: signs of a paper mill; suspected computer-generated content; unreliable results or conclusions; lack of ethics approval or compliance.

The experimental results showed that the injury mostly occurred in the knee joint, accounting for 33.4%, but the knee joint was mainly noncontact injury; the second was thigh injury, accounting for 8.5%. There were 3 cases of contact injury and 6 cases of noncontact injury; shoulder injuries occurred in 7 cases (6.3%); there were 2 cases of contact and 2 cases of noncontact in the head and face.

### 4.2. Injury Risk of Sports Competition under Multiple Algorithms

This experiment mainly investigated the relevant data of the six movements of treading, walking, jogging and standing long jump. Each movement lasts about 1 min, and the whole training process lasts about 10 min. During the training, relevant data are effectively recorded on the memory card. In the subsequent processing, the software automatically performs peak alignment and curve recording. The random forest algorithm is used to effectively classify the above data, and the error matrix is shown in Table 4.

Based on the error matrix of the table, the recall rates of random forest algorithm, machine learning algorithm and ant colony algorithm in the training set are further investigated. The experimental results are shown in Figure 5.

The results of the experiments demonstrate that as the number of experiments increases, the recall rate of the ant colony and machine learning algorithms also gradually rises. In this paper, only the random forest algorithm is comparatively flat. The recall rate of the machine learning algorithm reaches 0.66 when the number of experiments reaches 10, the recall rate of the ant colony algorithm reaches 0.62 and the recall rate of the random forest method is only 0.13. As a result, it can be said that the random forest algorithm has the lowest recall rate out of the three. Machine learning algorithm and ant colony algorithm are used for comparative analysis to show the performance of the monitoring system built by random forest algorithm. The length of time needed by the three classifiers to monitor damage is first looked into. The experimental results are shown in Figure 6.

The experimental results show that the random forest algorithm has the shortest training time among the three algorithms through the comparison of classifiers, and the testing time is close to 0S after the training, so the overall running efficiency is the highest. The machine learning algorithm adopts feed-forward approximation scheme, and the training and testing time is close, so it takes less time in small-scale testing, but the overall efficiency is not optimistic when the sample is further expanded. The training time of ant colony algorithm exceeds 0.7S, which is because the classifier of ant colony algorithm needs to measure the prior coefficients and weights, and the whole calculation process is complicated. The incidence of joint injuries corresponding to machine learning algorithm, ant colony algorithm, and random forest algorithm in this paper was compared with the actual incidence of joint injuries. 200 athletes were chosen as experimental objects.  Figure 7 displays the outcomes of a comparative experiment.

The article "Risk Management of Sports Venues and Olympic Sports Cooperation Spirit under Complex Environment" was retracted in 2023. Reasons: signs of a paper mill; suspected computer-generated content; unreliable results or conclusions; lack of ethics approval or compliance.

The experimental findings demonstrate that there is a significant difference between the incidence of joint injury under running intensity training as determined by machine learning and ant colony algorithms and the actual incidence of injury. The main reason for this is that, when the two methods mentioned above are used for injury analysis, it is challenging to analyse the influence mechanism of strengthening training load intensity on injury factors, which increases the deviation between the calculated incidence of joint injury and the actual incidence of injury. The change curve of joint injury rate obtained by random forest algorithm analysis in this paper is nearly identical to the change curve of the actual injury rate, demonstrating that the method suggested in this paper can analyse the influencing factors of joint injury with high fitting accuracy and that the analysis results are more accurate.

## 5. Conclusions

Sports industrialization, commercialization, and marketization all require effective risk management in the industry. This demonstrates how the sports industry has grown, with a major issue exposed in the growth being sports risk and the spirit of cooperation in Olympic sports. We should increase our understanding of problems and risk prevention in order to find problems, and we should perform well in precompetition project operation risk prevention, precompetition risk response and postcompetition liquidation evaluation. This paper investigates the spirit of Olympic sports cooperation and risk management of sporting venues using the random forest algorithm. The experimental findings reveal that the positions with the highest injury rates are the strikers, with an average of 54 injuries per striker, followed by defenders, with an average of 43 injuries per defender, and then the centre, with an average of 38 injuries per defender. Through the random forest algorithm, a special risk management organization is created prior to the event and is in charge of managing risks throughout the entire process, from planning to holding the event. A specialized risk management expert and a reputable insurance provider collaborate to develop and carry out the risk management plan, as well as to monitor and inspect it. It is necessary to analyse and study any risks that could jeopardize and affect the competition and the Olympic sports cooperation spirit through the random forest algorithm, as well as to fully prevent and deal with the risks. This will be the best opportunity to demonstrate to the world China's risk management capability of major sporting events and the Olympic sports cooperation spirit.

The article "Risk Management of Sports Venues and Olympic Sports Cooperation Spirit under Complex Environment" was retracted in 2023. Reasons: signs of a paper mill; suspected computer-generated content; unreliable results or conclusions; lack of ethics approval or compliance.

## Figures and Tables

**Figure 1:** Flow chart of decision tree growth process.

**Figure 2:** Sports injury monitoring system.

**Figure 3:** Damage between different positions on the field.

**Figure 4:** Participation in training during the preparation period.

**Figure 5:** Recall rate trend under three algorithms.

**Figure 6:** Comparison of training time of classifier under three algorithms.

**Figure 7:** Comparison of damage incidence among three algorithms.

**Table 1:** Results of average score of motor function and early injury.

	*N*	Mean ± SD	94% confidence interval	Percentage
History of injury	63	15.72 ± 2.62	15.05–16.38	88.55%
No history of injury	7	17.12 ± 1.25	16.17–18.06	11.42%

**Table 2:** Results of screening scores of motor function and symmetry of body.

	*N*	Mean standard deviation	94% confidence interval	Percentage
Body symmetry	22	17.31 ± 1.28	15.93–17.71	32.85%
Body asymmetry	46	12.95 ± 3.42	12.15–13.74	67.15%

**Table 3:** Statistics of injuries in the league preparation period.

position	Contact	Noncontact	Percentage
Head and face	2	2	2.4%
Shoulder	3	4	6.3%
Thigh	3	6	8.5%
Knee joint	8	21	33.4%

**Table 4:** Error matrix of random forest algorithm.

Activity	Stay where you are	Walk	Jogging	Standing long jump
Stay where you are	211	0	0	0
Walk	0	586	0	0
Jogging	0	0	95	0
Standing long jump	5	6	2	147

## Data Availability

The data used to support the findings of this study are available from the author upon request.
